The article "Construction of a Ceramic Appearance Design System Based on Technology for Internet of Things" was published in 2022. Journal: Comput Intell Neurosci.

# Construction of a Ceramic Appearance Design System Based on Technology for Internet of Things

**DOI:** 10.1155/2022/7490051

**Published:** 2022-05-17

**Authors:** Zhou Long, Junzhe Ouyang

**Affiliations:** ^1^Art and Archeology School, Jingdezhen Ceramic University, Jingdezhen, Jiangxi 333403, China; ^2^Library, Jingdezhen Ceramic University, Jingdezhen, Jiangxi 333403, China

## Abstract

The planning and design of intelligent storage systems in ceramic parks based on the industrial Internet of Things technology are proposed. Based on the analysis of the storage demand of ceramic parks, information transformation is carried out according to the original manual operation mode. The RFID technology is applied to the overall planning of the warehouse area and the deployment of the software; it is applied to the overall planning of the RFID system, the hardware deployment of the two-dimensional warehouse system, and the integration of the RFID technology and the software deployment of the two-dimensional warehouse system. It realizes the close cooperation between the information system and hardware equipment, optimizes the system process, and improves the level of warehouse management.In addition, smart terminal ceramics refer to those with fine ceramic appearances or functionalities in smart terminal products, such as smartphones, smart watches, and other wearable devices, in the field of consumer electronics, including ceramic back plates, middle frames, buttons, fingerprint recognition sheets on mobile phones and ceramic cases, bracelets, and back covers on smart watches. Aside the excellent performance and aesthetic properties of ceramic materials, they can also be adapted to the trends in 5G and wireless communication technology. From the perspective of high strength, high toughness, and colorful nano-zirconia ceramics, this article was aimed to review the development process and industrialization application process.

## 1. Introduction

With the impact of the wave of “industry 4.0” and “intelligent manufacturing,” all enterprises are carrying out the work of improving the manufacturing level of enterprises, especially improving the logistics system [1], which is the weakest link in the process of enterprise production management. The production process of ceramic products is complex and there are many kinds of products. The finished products and semifinished products mostly exist in the form of solid and solid-liquid mixture, and the raw materials are flammable, explosive, and toxic. Therefore, there are more strict requirements for the storage of products and raw materials [2]. There are differences in grade, color number, and size of products, which are uncontrollable, resulting in the production personnel not knowing the specific situation of each batch of products, often resulting in the decline of the rate of high-quality products. Some ceramic enterprises use pure manual operation to record the operation of logistics process through paper forms [3]. Some companies are also using 1D barcode technology to manually scan barcodes to record goods entering and leaving the warehouse. When the goods are in and out of the warehouse, it is necessary to stop logistics and wait for scanning [4–6]. The scanning workload is heavy, and there may be missed scanning, repeated scanning, and other situations, resulting in low scanning efficiency. In addition, in ceramic enterprises, products have different specifications such as boxes and bags, which also makes it difficult to build ceramic warehousing and logistics systems [7]. Therefore, relevant experts in the ceramic industry and logistics industry are carrying out relevant technology application research. Using the system structure platform of the industrial Internet of Things, the research on the establishment of a third-party supply chain management platform is carried out by upgrading and integrating technical means such as the bar code technology, the RFID technology, the GPS/GTS technology, and Internet technology [8, 9]. In addition, smart terminal ceramics generally refer to various precision ceramic materials and appearance structural parts used in smart terminal products in the field of consumer electronics. Smart terminal products mainly include smartphones, smart watches, smart bracelets, smart glasses, and other wearable devices. Precision ceramic parts used in smartphones include mobile phone ceramic backplanes [10], ceramic middle frames [11], ceramic keys [12, 13], fingerprint identification ceramic chips [14], etc., as well as single crystal alumina (sapphire) and transparent ceramics for mobile phone display screens. The applications in smart wear include ceramic watch cases, ceramic watch chains, and ceramic back covers on smart watches, as well as appearance ceramic parts on smart bracelets and necklaces [15]. Therefore, it can be said that intelligent terminal ceramics integrate the functional, aesthetic, and artistic characteristics of ceramic materials.

In this paper, based on the analysis of the current situation of warehousing in a ceramic park, a system architecture based on the industrial Internet of Things is proposed, combining the RFID technology with the two-dimensional barcode technology to intelligently transform the original warehousing system, which not only solves the system cost problem, but also solves the problem of reading and writing wireless information.

## 2. Application Requirements of Ceramic Storage

### 2.1. Storage Status of a Ceramic Park

A ceramic park has a large-scale, wide geographical distribution and frequent goods in and out. A manual forklift operation is adopted for warehousing. Manual warehousing, inventory, and other operations are carried out, and relevant information is recorded in the account manually. At the same time, the goods are stacked disorderly.

With the development of the times and the progress of technology, the existing model can no longer meet the needs of rapid social development:

1. Slow logistics turnover in the park
2. In this paper, the multi-sheet method is adopted for vehicles entering and leaving the factories in the park. The driver needs to go to multiple departments, and the property management personnel also need to input and transfer various data in order to complete the relevant procedures of entering and leaving the factory, which directly leads to the slow logistics turnover in the park.
3. Inefficient warehousing operation
4. Warehousing operations such as purchase, delivery, selection, and inventory are completely managed manually. In some factories, inventory is made once in daily inventory.
5. The library needs 3 people and takes nearly 1-2 days. It is not only inefficient, but is also prone to human errors.
6. Information cannot be shared and data are entered repeatedly
7. The manual input of vehicle license plate and floor weight increases the efficiency of manual data entry, which reduces the manual input of vehicle license plate, floor weight, and other related data.
8. Unable to grasp the production and operation in time
9. Due to the existence of information island, the Storage and Transportation Department of the supply chain center cannot timely obtain the inventory information of raw materials, semifinished products, finished products, and other manufacturing factories, cannot grasp the overall inventory of the enterprise in real time, and the enterprise management and employees cannot grasp the relevant information in the production process.
10. One-dimensional bar code data loss and inaccuracy
11. In many factories, a one-dimensional bar code technology may be used for storage, but the amount of one-dimensional bar code information is too small, which is prone to physical damage, the system cannot be entered, and the data are lost. Therefore, a contactless way of information storage is needed.  Figure 1 shows the ceramic hardware architecture.

### 2.2. Storage Development Direction of a Ceramic Park

1. Use RFID, big data, cloud computing, and other technologies to design the inventory management system, post RFID tags on finished products, semifinished products, raw materials, and other inventory items [16], and build the system structure based on the industrial Internet of Things(see Figure 2)
2. Build a three-dimensional warehouse, explore the storage capacity resources in space, plan the combination of semiautomatic equipment and software system, improve the real-time inventory information of materials, and accelerate the speed of material turnover
3. Realize the two-dimensional coding of products, support fast code scanning of warehousing operations, and speed up warehousing and subsequent traceability
4. Get through the communication links of Weighbridge and quality inspection, and share the weighing and quality inspection data
5. Replace experience with technology to improve the overall informatization level of warehousing in the park

## 3. Intelligent Terminal Ceramic and 5G Communication and Wireless Charging

In recent years, smart terminal ceramics have developed rapidly and received high attention from the market, mainly because precision ceramic materials have some excellent properties and characteristics that other smart terminal materials (such as metal and plastic) do not have, and can meet the development trend of 5G communication and wireless charging.

With entering the 5G era, as 5G communication adopts wireless spectrum above 3 GHz, the antenna structure of smartphones will be more complex than 4G, with greater signal transmission volume and faster transmission speed. At present, the aluminum-magnesium alloy widely used in mobile phone shells cannot meet the requirements of 5G signal transmission and wireless charging because of its strong signal shielding effect [17]. However, ceramic materials have small signal shielding, which is convenient for wireless charging, and the antenna structure is easy to design.

Wireless charging technology is mainly realized by magnetic resonance, electric field coupling, magnetic induction, and microwave antenna transmission technology. At present, the metal casing can shield and absorb the electromagnetic field, which will affect the transmission efficiency of wireless charging; thus, the wireless charging function cannot be used in metal back covers for mobile phones and smart watches.

However, electromagnetic waves can smoothly pass through non-metallic materials such as ceramics, glass, and plastics. Therefore, in order to realize the wireless charging function of smartphones and watches, ceramic and glass back covers must be used. Although plastics can also be used, they are easy to age and have poor texture. As can be seen, ceramic materials are a better solution to signal transmission problems, both for 5G communication and wireless charging.  Figure 3 illustrates the business flowchart of ceramic production.

It has the advantages of good wear resistance and anticorrosion of zirconium, and it is not comfortable to wear on the skin. Thus, it is more suitable for intelligent wearable devices. As early as 2015, when the Apple watch was launched, nano-zirconia ceramic material was used as the back cover of smart watches for the first time to facilitate wireless charging. This black circular zirconia ceramic back cover was mainly produced and provided by Lansi Technology Co., Ltd. Subsequently, in 2016, Apple released the precision ceramic Apple watch Edition 2, which has a magnetic suction wireless charging base and a charging head of 5via [18–20]. In 2016, Huami technology, the manufacturer of Xiaomi watch, took the lead in launching the first all-ceramic bezel sports watch of Amazfit brand and the later Amazfit smart sports watches. The bezel adopts zirconia ceramics.

High-tech ceramics have become an indispensable element of Huawei smart watches. At the press conference at the end of 2018, Huawei launched the dark blue ceramic version of the glory watch magic series and the dream quicksand apricot ceramic version. It selected the industry-leading 3D curved surface ceramic precision machining technology to create a ceramic bezel through multiple processes. Among other things, the quicksand apricot ceramic plate is made of nano-zirconia powder and spinel high temperature-coloured ionic oxide. After high-temperature sintering, it turns pink and soft apricot colors.

In recent years, glass backplane has also been widely used in smart phones, such as iphone 8, Samsung note8/S8, glory 9, Xiaomi 6, and other brand phones. The advantages of a glass body mainly lie in avoiding the shielding of mobile phone signal, good texture, and hand feel, but because glass is a kind of amorphous material of silica, it is easy to break and scratch. Corning, the world's largest supplier of mobile phone glass, has launched the fifth generation of gorilla glass. Although its strength has been improved, its hardness is still not as good as sand and is prone to scratches. In addition, glass processing is more difficult than metal, especially arc surface and mobile phone middle frame. At the same time, tempered glass can easily fracture to form a striped fracture crack path, which can easily cause edge collapse.

The bending strength of Y-TZP nano-ceramics with rare earth Y2O3 as a stabilizer is usually more than 1000 MPa, which is greater than that of glass back plates. The fracture toughness is also twice that of glass. The elastic modulus and Vickers hardness are much higher than that of glass, which are 210 GPA and 1300 HV, respectively, while for Corning glass they are only 50 GPA and 583 HV. Obviously, the wear resistance and scratch resistance of ceramics are better than that of glass. Figure 4 illustrates the relationship between deviatoric stress and normal strain of ceramic products.

In terms of structural design, under the same strength, the ceramic back plate is thinner than glass, which can be reduced by about 40%, leaving more space for the structural design of mobile phones [21]. In addition, the surface of ceramic backplanes can be processed to obtain a variety of surface effects, such as bright, matte, wire drawing, and other mechanical textures. The surface can also be changed through laser, mcvn, PVD silk screen printing, painting and edge C angle, R angle, and other processes. In particular, the nano-zirconia ceramic back plate has a diamond-like shine and jade-like warmth, displaying its elegance and unique charm.

## 4. Overall System Planning

For the architecture of a warehousing and logistics system based on industrial Internet of Things, the whole scheme should be considered to define system standards around the three themes of “IOT perception,” “data collaboration,” and “platform management,” so as to build an upper management or supervision platform and a lower control platform. In this system, RFID tags will be posted on any items to be stored or raw materials, and each tag has a unique identification (ID), including item code and product batch, so as to realize IOT perception. At the same time, the system also needs to realize the interconnection between the data system and handheld devices, forklifts, AGVs, and other equipment. The tag is scanned by the RFID reader. After scanning, the reader extracts the ID of the tag and transmits it to the platform management layer. The platform management layer uses big data and cloud computing technologies to receive the reader location, reading time, and read data. Based on these data, cloud computing will use the corresponding ID to point out the location and visualization results of items, and display the real-time data and real-time updates of the movement of inventory items to users, so that enterprise employees can use smartphones or laptops to monitor the inventory in real time from anywhere. The overall structure of the system and handmade ceramic products is shown in Figure 5. WMS, warehouse management software, is an essential core management software in warehouse logistics systems. It is an intelligent and lean warehouse management system designed to solve the problem of extensive management of ceramic parks. The system interacts with ERP, MES, TMS, LIMS, and other systems through data interface. With data interfacing, data collection can effectively solve the situation of each system working in isolation.

WMS takes barcode and RFID as the information cornerstone for business operations such as warehousing, outbound and in-warehouse operations of warehouse items, and realizes the functions of real-time scheduling of business operations, information release, prompt and operation guidance, operation result data return, delivery, historical operation information tracking, and so on, so as to achieve high visibility, high controllability, and high accuracy of the warehouse operation process for the purpose of being highly traceable.

In order to achieve the goal of intelligent and lean warehouse management, the intelligent warehouse system is deployed from the aspects of platform reservoir area planning, identification planning, warehouse location design, RFID and QR code equipment deployment, system architecture design, system business process implementation, software platform, and so on.

### 4.1. Platform Reservoir Area Planning

According to the characteristics of the ceramic park, different buildings need relevant planning, including platform reservoir area, platform, high shelf area, etc., as follows:

1. Platform reservoir area planning
2. Generally speaking, the ceramic park is composed of multiple factory warehouses and several logistics warehouses. Although the materials stored in each warehouse are different, each warehouse will have a platform (buffer area) for the preparation of materials in and out of the warehouse. The introduction of shelves makes the use and management of the warehouse extremely beneficial.
3. Platform planning
4. Platforms can be divided into unloading platforms, loading platforms, and common platforms according to their functions. In order to save space and improve the utilization of the platform, the platform is planned as a common platform.
5. High shelf area planning
6. The shelf area of the warehouse in the ceramic park is used to store goods or raw materials with pallets as containers. The shelf area can be further divided into qualified product area and unqualified product area according to the attribute of goods. According to different product raw materials, it can be divided into raw material area, semifinished product area, and finished product area.

### 4.2. Material Identification Planning

In order to realize the fine management of the warehouse, the intelligent storage system must uniquely identify the items, location, and pallet in the warehouse. The unique identity has two meanings:

1. The attribute information of items, storage locations, etc., can make intelligent devices (RF equipment or bar code equipment) with fast identification and uniqueness.
2. Items, warehouse location, and other information can enable operators to quickly identify. In order to achieve the above two functions, the items and storage space identification are divided into equipment identification and personnel identification. For the equipment identification mark, the system adopts the combination of the RFID identification technology and 2D barcode to collect information.

There are equipment identification, personnel identification, and overall design drawing of ceramic warehouse. For equipment identification, the system adopts a combination of the RFID technology and two-dimensional bar code to collect information.

The personnel identification sign is mainly through the production of eye-catching signboards, so that the operators can quickly see the required information, as shown in Figure 6.

### 4.3. Location Design

1. Elevated storage location design
2. In order to facilitate the warehouse location management and operation, the intelligent storage system can quickly guide the operators to lock the warehouse location, configure one two-color tower lamp for each shelf, one RFID tag and one warehouse location bar code for each warehouse location, identify the layer column number of the warehouse location on the warehouse location, and stick the warehouse location code on the shelf column, as shown in Figure 6.
3. Plane location design
4. Depending on the characteristics of the ceramics business, many raw materials and finished products are stored in a flat warehouse. In order to effectively control the stacking area, the intelligent warehouse plans the flat storage area into several locations, pastes the location bar code on each location in the stacking area (the location bar code needs to include the row and column coordinate parameters of the location, so that the operators can quickly lock the location), and pastes the material bar code on the material barrel or bag. When entering the warehouse, the operators bind the materials and location information by scanning the material bar code and location bar code, so as to realize the lean management of materials and storage area. The histogram of ceramic content and ceramic stress ratio is as shown in Figure 7.

### 4.4. RFID and QR Code Equipment Deployment

1. Tray label
2. The label is installed on the side or above the pallet in a non-cargo-sheltered position. The label can be pasted and installed, and the appropriate installation method can be selected according to the situation of the tray.
3. Forklift reader
4. The RFID reader is installed at the lower end of the front of the forklift, and the active reader is installed at the rear end. The reader can be fixed by rivets or screws. Variation curves of pore pressure of ceramic products with stress levels are shown in Figure 8.
5. Installation of door and entrance label
6. According to the actual situation, install the label at the upper end or side end of the inner side of the warehouse door. The label can be hung or pasted.

## 5. Preparation Technology of Intelligent Terminal Ceramics

The preparation technology of ceramic powder in the middle section includes the preparation technology of ceramic powder in the front section and the polishing technology of ceramic parts in the middle section. These three technologies directly affect the material properties and product quality of various forms of intelligent terminal ceramics.

### 5.1. Preparation Technology of Nano-Ceramic Powder

The previous process is mainly the synthesis and preparation technology of high-performance nano-zirconia powder. In order to give consideration to the good strength and toughness of the material, this kind of nano-zirconia powder usually introduces 2 mol%–3 mol% rare earth yttrium oxide (Y2O3) as the stabilizer, so as to obtain the nano-zirconia powder with metastable tetragonal zirconia as the main crystal phase, which has no agglomeration/impurities. The sintering activity is good, and the sintered material has high bending strength, fracture toughness, and good fall resistance. Specifically, the powder requires appropriate and uniform chemical composition, good dispersion state, appropriate grain size, appropriate specific surface area, and appropriate phase composition.

In addition, the preparation technology of color zirconia ceramic powder is becoming more and more mature. By introducing different colored oxides or colored ions in the process of powder synthesis, including oxide coloring and spinel coloring, zirconia ceramic powders with dozens of colors can be obtained. The color series that Chaozhou Sanhuan can mass produce on the ceramic back plates of mobile phones includes Tiffany blue, Morandi grey, Shuihu blue, cherry powder, violet, dark blue, and Porsche grey. These colors mainly come from luxury brands, such as Tiffany and Porsche, which lead the modern trend and fashion, and have a strong sense of science and technology. In addition, malachite green inspired by Dunhuang murals and Ji blue-glazed zirconia powder from the Xuande era of Ming Dynasty collected by the Forbidden City have also been developed and applied to Xiaomi mix2s emerald ceramic edition mobile phones and Xiaomi mix3 Imperial Palace sapphire blue ceramic collection mobile phones in 2018, respectively.

The colorants of zirconia ceramics are mainly ionic crystal compounds, and the coloration ions are usually transition metal ions and rare earth metal ions. The transition metal ions have 4s1-23dx electronic structure, and the rare earth metal ions have 6s1-25d1-84fx electronic structure. Their outermost S-layer, sub-outer D-Layer, and even the F layer of the third layer calculated inward from the outermost layer are not filled with electrons. These unpaired electrons are unstable and easy to transition between the sublayers of each layer.

At present, spinel-type pigments, perovskite-type pigments, and silicate-type pigments are widely used in color zirconia ceramics in intelligent terminals. In particular, spinel-type pigments have excellent properties such as high-temperature resistance, strong atmosphere change resistance, and good chemical stability. They are not easy to decompose and color stably and brightly in the high-temperature (1350°C–1500°C) densification and sintering process of zirconia ceramics. The results show that the microstructure of white 3Y-TZP ceramics sintered at atmospheric pressure has a grain size of about 350 nm, which has a wide application prospect. This is the same as the microstructure of blue zirconia ceramics. It can be observed that the colored spinel CoAl2O4 phase is distributed in zirconia grains, and a clean grain boundary is formed between zirconia grains.

### 5.2. Forming and Sintering Technology of Ceramic Products

Mobile phone ceramic backplane molding process mainly includes dry pressing + cold isostatic pressing, injection molding, gel casting, and casting + warm compaction hot bending—four kinds of molding methods.

1. Dry pressing + cold isostatic pressing
2. The process is a spherical particle of ceramic powder after spray granulation (particle size 50 *μ*m–200*μ*m). Firstly, the ceramic back plate blank with a regular shape of 2.5*D* or 3*D* is obtained by pressing and forming in the metal mold. Then, it is put into the rubber mold and vacuum wrap before passing through 150 MPa–200 MPa Cold Isostatic Pressing (CIP) treatment, which greatly improves the density, strength, and uniformity of the ceramic back plate blank, which is conducive to ensuring the consistency and reliability of mechanical properties and microstructure of sintered products. This forming process has the advantages of uniform product density, high strength, and small sintering deformation. In particular, ceramic products are virtually free of air and pinholes after grinding and polishing. It has become one of the mainstream forming technologies for ceramic back plates for mobile phones.
3. Ceramic injection molding
4. The process is to heat and mix ceramic powder with high molecular binder (such as polyethylene, polypropylene, polyformaldehyde, and polystyrene) and low molecular plasticizer, dispersant, and lubricant (such as paraffin and stearic acid) in an internal mixer, then granulate with a granulator, and obtain ceramic blanks with various complex shapes through injection molding with a special injection machine. The organic additives in the blank are discharged through the degreasing and degumming process (such as thermal degreasing, solvent extraction degreasing, and catalytic degreasing), and finally densified sintering is carried out.  Figure 9 shows the photos of the ceramic back plate and middle frame of mobile phones prepared by injection molding before and after degreasing and sintering.
5. Injection molding is especially suitable for the manufacturing of wearable ceramic appearance parts such as 3D-shaped ceramic cover plates and smart watches. Due to the high degree of automation in the forming process, it facilitates efficient mass production, high-dimensional accuracy of the formed blanks, and less processing after sintering, which helps reduce processing costs. It has become the mainstream molding technology of smart ceramic watches and ceramic bracelets.  Figure 9 shows the ceramic watch ring smart watch designed by Huawei Watch GT 2 Porsche, and it shows Xiaomi's Amazfit “equator” and “moon frost” ceramic bracelets.
6. Gel casting process
7. The process introduces organic monomers and crosslinking agents into the ceramic slurry, adds the initiator and catalyst, and then uses non-porous mold (such as metal, glass, and plastic) for pouring molding. The slurry in the mold is solidified through the polymerization reaction of organic monomers to obtain the 3D or 2D ceramic blank with the required shape. The formed blank has high strength and less organic binder content. This technology was applied to the forming and preparation of 2D ceramic backplanes of Huawei P7 Collection Edition in the early stage, and molar circle and shear strength envelope of ceramic products, as shown in Figure 10. However, the low level of mechanisation and efficiency makes it difficult to control the consistency and stability of the product during the forming process. At present, it has not been widely used in the forming of ceramic appearance parts of intelligent terminal.

## 6. Business Process Optimization

### 6.1. Optimization of the Receiving Management Process

When the freight vehicle arrives at the unloading area, it enters the goods receiving link, which is the preparation link of goods warehousing. The effective stress path curve of different ceramic contents is shown in Figure 11.

The intelligent warehousing system obtains the warehousing notice from the ERP system through the interface (there are many types of warehousing notices, such as finished product warehousing notice, purchase warehousing notice, return warehousing notice, replenishment warehousing notice, etc.), and the management personnel create the warehousing notice based on the warehousing notice combined with the items that need to be warehoused this time.

The operators check and inspect the goods according to the warehousing order, and feed back the results to the WMS software, which prints the bar code of the goods. If the goods need to be stored on a pallet, the barcode information of the goods needs to be bound with the pallet after the goods are pasted. The WMS software generates an inbound task upon receipt of feedback and the operator performs the inbound operation upon the receipt of the task.

The specific process of receiving is as follows.

When creating a receipt document, managers should choose whether there is a need for quality inspection. Quality inspection in the receiving phase is an optional function. If the operator does not select quality inspection, the receiving phase only needs to check the quantity and category of goods.

When the goods arrive at the platform, the warehouse personnel will check and visually inspect the goods according to the warehouse receipt. After passing the visual inspection, the warehouse personnel will enter the article name, supplier name, article batch information, article production date, material content, actually received quantity, and quality inspection results in the system (if there is such information in the warehouse receipt, it is unnecessary to enter it).

Operators unload the same kind of goods at one time. After unloading, they stack and support the goods of the same type and batch. The WMS software generates cargo barcodes based on the incoming order information and manually enters cargo information, the system prints labels and manually pastes the codes on-site, binds the cargo information to the pallet, and then receives the next type of cargo.

### 6.2. Optimization of the Warehousing and Shelving Process

After the goods are received, the WMS software recommends the storage location for all the goods to be warehoused this time according to the storage location strategy, and assigns operators to the warehousing operation according to the article properties or the area where the article storage location is located. The operator receives the operation task and scans the forklift bar code or the RFID tag with the handheld operation terminal to bind the forklift to the operator (the second scan will be unbound or the operation task completion system can also be unbound automatically). If not, the system will give an alarm. When the operator starts the warehousing task, the system lights up the indicator light of the roadway where the warehouse location needs to be put on the shelf in this warehousing task into red, displays the warehouse location information on the computer, and guides the forklift to quickly and accurately lock the warehousing location through the on-board computer and the roadway tower light.

After the forklift arrives at the assigned warehouse location of the system, the on-board RFID scans the warehouse location label to confirm whether the warehouse location is correct (misreading needs to be considered here). If the goods are put on the shelf correctly, confirm that the putting on the shelf is completed. If the warehouse location is wrong, look for the correct warehouse location. If the location label fails or the on-board RFID fails, the location can be confirmed by hand scanning the location barcode. The WMS software will update the location information after the shelf is completed. If the location is full, the system will mark the location status from idle to occupied. In the subsequent shelf location allocation, the location will no longer participate in the location allocation (the intelligent storage system will consider the capacity of the location, and may recommend it again if the location is not satisfied). After all warehousing operations are completed, turn off the roadway indicator tower light. The intelligent storage system is put into storage and put on shelves through lighting and on-board. Computer guidance makes the storage and shelving process fast. At the same time, the WMS software can identify items that do not belong to the task of this operation through the error-proof function of the access control, thus making the storage and shelving process accurate.

## 7. Conclusion

Based on the industrial Internet of Things technology, the intelligent storage system of the ceramic park realizes the functions of cross-regional centralized management, distributed operation, and real-time monitoring, and can efficiently complete various business operations. By improving the storage management, the identification rate of goods in and out of the warehouse is improved, multiple goods can be identified at the same time, so as to ensure the consistency between the quantity of physical goods and documents, and the efficiency of in and out of the warehouse process improved. It also reduces the counting cycle, realizes real time and dynamic grasp of inventory, and visual management of inventory items. By accurately mastering the inventory situation, we can optimize the reasonable inventory, understand the status and changes of the warehouse environment in real time, observe the work situation of the staff in the warehouse in real time, and understand the work progress. Through RFID, big data, cloud computing, and other technologies, the smart storage system realizes the close cooperation between the information system and hardware equipment, optimizes the system process, and improves the work efficiency of the supply chain management department of the ceramic park. In addition, the nano-crystal zirconia ceramic material is adopted, and the seamless connection between the ceramic back plate and the metal middle frame makes it light and moist as jade as a whole. Its hardness is close to sapphire, but its bending strength and fracture toughness are much higher than sapphire crystal. It has excellent wear resistance, durability, silky feel, and the surface is as clear and shining as diamond after grinding and polishing. With the advent and popularization of 5G, the metal back plate of mobile phones will gradually withdraw, and the ceramic back plate will occupy a larger market share.

## Figures and Tables

**Figure 1:** Ceramic hardware architecture.

**Figure 2:** Overall planning of the ceramic warehouse system.

**Figure 3:** Business flowchart of ceramic production.

**Figure 4:** Relationship between deviatoric stress and normal strain of ceramic products. (a) Ceramic casting pressure 100 kPa. (b) Ceramic casting pressure 200 kPa.

**Figure 5:** Photos of handmade ceramic products.

**Figure 6:** Overall design drawing of a ceramic warehouse.

**Figure 7:** Histogram of ceramic content and ceramic stress ratio.

**Figure 8:** Variation curve of pore pressure of ceramic products with stress levels. (a) Ceramic casting pressure 100 kPa. (b) Ceramic casting pressure 200 kPa.

**Figure 9:** Flowchart of ceramic shelves.

**Figure 10:** Molar circle and shear strength envelope of ceramic products.

**Figure 11:** Effective stress path curve of different ceramic contents. (a) Ceramic casting pressure 100 kPa.  (b) Ceramic casting pressure 200 kPa.

## Data Availability

The data used to support the findings of this study are available from the corresponding author upon request.
